# The Difference between Sacubitril Valsartan and Valsartan on Vascular Endothelial Function, APN, MMP-9, and BNP Levels in Patients with Hypertension and Chronic Heart Failure

**DOI:** 10.1155/2022/9494981

**Published:** 2022-02-18

**Authors:** Haiping Du, Xiao Li, Weifang Zhao, Ning Jiang

**Affiliations:** ^1^Department of Cardiology (I), East Hospital, Yantaishan Hospital, Yantai 264000, Shandong, China; ^2^Department of Cardiology (II), The Third People's Hospital of Qingdao, Qingdao University, Qingdao 266041, Shandong, China; ^3^Cardiac Function Examination Room, Affiliated Qingdao Central Hospital, Qingdao University, Qingdao 266042, Shandong, China; ^4^Department of Hypertension, Jinan Municipal Hospital of Traditional Chinese Medicine, Jinan 250012, Shandong, China

## Abstract

**Background:**

Sacubitril valsartan and valsartan are the first new drugs approved for angiotensin receptor neprilysin lysine inhibitors (ARNIs) in outpatients with chronic heart failure (CHF) and hypertension. Compared with enalapril, sacubitril valsartan and valsartan have been shown to reduce the mortality and morbidity of cardiovascular diseases. However, there is little actual evidence regarding the efficacy of ARNIs in hypertensive patients with CHF.

**Methods:**

From January 2019 to January 2021, 60 patients with hypertension and chronic heart failure were diagnosed and treated in our hospital. The patients were randomly divided into an observation group and a control group, with 30 cases in each group. The control group was given valsartan, the observation group was given sacubitril valsartan, and both groups were treated for six months. The endothelium-dependent vasodilation (EDD) function of the brachial artery and serum nitric oxide (NO), endothelin-1 (ET-1), carotid artery intima-media thickness, and glomerular filtration, excess rate (eGFR), and left ventricular ejection fraction (LVEF) were compared between the two groups of patients before and after treatment. The serum adiponectin (APN), matrix metalloproteinase-9 (MMP-9), and brain natriuretic peptide (BNP) levels were compared before and after treatment.

**Results:**

The total effective rate of treatment in the research group was higher than that in the control group (*P* < 0.05). After treatment, the cardiac function indexes LVESD and LVEDD of the two groups of patients were lower than before treatment, and LVEF was higher than before treatment, and the improvement rate of the treatment group was better than that of the control group (*P* < 0.05). After treatment, the serum APN of the two groups was higher than before treatment, the levels of MMP-9 and BNP were lower than before treatment, and the improvement rate of patients in the treatment group was better than that of patients in the control group (*P* < 0.05). There was no statistically significant in the levels of EDD, NO, and ET-1 of the two groups of patients before treatment (*P* < 0.05). After treatment, compared with the control group, the EDD function and NO level of the research group were significantly increased (*P* < 0.05), and the level of ET-1 was significantly reduced (*P* < 0.05). There was no statistically significant difference in carotid artery intima-media thickness, glomerular filtration rate, and left ventricular ejection fraction before and after treatment in the two groups (*P* < 0.05).

**Conclusion:**

In the treatment of hypertension and chronic heart failure, sacubitril valsartan can improve the clinical symptoms of patients to the greatest extent and can significantly improve the levels of LVEF, LVEDD, NT-proBNP, heart function, and other indicators. Sacubitril valsartan can increase serum APN levels, reduce MMP-9 and BNP levels, and have good clinical effects. Sacubitril valsartan has a protective effect on the vascular endothelial function of patients with hypertension and CHF. However, these results need to be confirmed in studies involving more subjects and require longer follow-up times.

## 1. Introduction

Chronic heart failure (CHF) is one of the common diseases in cardiology. Chronic heart failure is mostly caused by a variety of factors that lead to changes in the structure and function of the heart, causing ventricular contraction and/or diastolic dysfunction so that the cardiac output cannot meet the metabolic needs of the body, thereby causing cardiac circulatory disorders [1]. In recent years, due to changes in dietary structure, the number of people with high blood pressure in my country has gradually increased, reaching 27.1% [2], and long-term uncontrolled high blood pressure can lead to CHF. At present, despite the continuous improvement of CHF treatment, its 5-year survival rate is still low [3, 4]. In the occurrence and development of CHF, its vascular endothelial dysfunction and the disease itself are mutually causal. Endothelial dysfunction leads to an imbalance in the levels of NO and ET-1 released by endothelial cells, resulting in abnormal vasomotor function, which further leads to increased vascular resistance and increased cardiac afterload, thereby aggravating myocardial ischemia and hypoxia, pumping dysfunction, and forming a vicious circle [5–7].

An important feature of the pathogenesis of hypertension and chronic heart failure is the activation of the neurohormonal system, including the renin-angiotensin-aldosterone system (RAAS) and the sympathetic nervous system (SNS). In the short term, the compensatory activation of these systems is conducive to increasing blood pressure and enhancing cardiac contractility, which stems from their evolutionary “biological protection” role. However, the continuous excessive activation of these systems often produces the opposite effect, inducing and aggravating cardiovascular disease and worsening heart failure due to fluid retention [8]. Based on the understanding of its mechanism, drugs that inhibit these neurohormonal systems have been shown to be used to treat cardiovascular diseases, such as hypertension and heart failure, and can reduce the mortality and hospitalization risk of heart failure by 37% [9]. Therefore, it is particularly important to choose a reasonable and effective treatment plan for patients with hypertension and chronic heart failure.

Sacubitril valsartan and valsartan are angiotensin receptor-enkephalinase inhibitors (ARNI), which can simultaneously inhibit RAAS and regulate NPS, promote water and sodium excretion, dilate blood vessels, and antagonize sympathetic activity. At the same time, sacubitril valsartan and valsartan have anti-inflammatory, antiventricular remodeling, and antihypertensive effects, thereby improving the treatment effect and prognosis of patients [10–12]. Therefore, sacubitril valsartan and valsartan are approved as first-line treatments to reduce heart failure [13]. Clinical trials have confirmed the effects of sacubitril valsartan and valsartan in improving heart failure and revealed their potential in blood pressure control [14, 15]. Studies have shown that it is easier to improve the prognosis in patients with CHF than angiotensin-converting enzyme inhibitors (ACEI) [16, 17]. Sacubitril valsartan sodium is mainly used clinically to treat chronic heart failure with reduced ejection fraction. Sacubitril valsartan sodium inhibits enkephalinase through the active metabolite of the prodrug sacubitril and, at the same time, block the type 1 receptor of angiotensin II by valsartan, thereby improving the prognosis in patients with chronic heart failure [18].

This article explores 60 patients with hypertension and chronic heart failure, adopts the clinical efficacy of two treatments, provides a more clinical application basis for the adjustment of blood pressure level, and provides better guidance for clinical work. This study aims to further explore and analyze the effects of valsartan and valsartan treatment of sacubitril on vascular endothelial function, APN, MMP-9, and BNP levels in patients with hypertension and chronic heart failure based on previous research.

## 2. Material and Methods

### 2.1. Research Object

A total of 60 patients with hypertension and chronic heart failure who were diagnosed and treated in our hospital from January 2019 to January 2021 were selected and randomly divided into a research group and a control group. The patients were randomly grouped, and the patients were numbered according to the sample size, from 1 to 60, and random numbers were generated using SPSS26.0. Starting from any number in the random number table, take a random number for each research subject in sequence along the same direction. Thirty patients with a larger random number were used as the research group, and 30 patients with a smaller random number were used as the control group. This study was conducted after being approved by the ethics committee of our hospital.

Inclusion criteria were as follows: meeting the diagnostic criteria for hypertension; patients aged ≥18 years; patients with chronic heart failure whose heart function is graded II-IV by NYHA; patients who have good compliance and can be followed up in time. The patients and their families have been informed of the purpose and methods of this study, and their right to informed consent is reserved.

Exclusion criteria were as follows: patients who are allergic to all the ingredients of the drug or its active ingredients (sacubitril valsartan) or any excipients; patients with angioedema (whether hereditary or idiopathic); patients with severe liver function impairment; patients with biliary cirrhosis and cholestasis; patients with severe renal impairment (GFR <30 ml/min), serum potassium >5.4 mmol/L; patients in the second and third trimesters of pregnancy; diabetic patients who also used aliskiren; patients with systemic diseases such as tumors and immune systems; patients who refused to continue to participate in the study and who were lost to follow-up.

### 2.2. Research Methods

#### 2.2.1. Treatment Methods

All patients undergo routine treatment and care for chronic heart failure and hypertension, including limiting salt intake, proper diuresis, oxygen inhalation, correcting electrolytes, and application of drugs (*β*-blockers, vasodilators). On the basis of conventional treatment, patients in the control group chose valsartan capsules (National Medicine Standard H20040217, the specification is 80 mg/capsule) 80 mg/time, twice a day. The research group added sacubitril and valsartan sodium tablets (Beijing Novartis Pharmaceutical Co., Ltd., specification 100 mg, National Standard H20170343) 50 mg/time on the basis of conventional treatment, twice a day. According to the tolerance, sacubitril and valsartan sodium tablets are increased to 100 mg/time, two times a day, orally. The blood pressure control goals of the two groups of patients were systolic blood pressure <130 mmHg and diastolic blood pressure <80 mmHg. If the blood pressure control target cannot be achieved, additional drug doses or combined application of other drugs can be used if necessary.

### 2.3. Evaluation of Detection Indicators and Clinical Efficacy

#### 2.3.1. Criteria for Clinical Efficacy Evaluation

Significantly effective: the clinical symptoms and signs of the patient such as dyspnea, fatigue, and edema were significantly improved compared to before treatment, and the NYHA cardiac function classification improved to 2 or more. Effective: the patient's clinical symptoms and signs such as dyspnea, fatigue, and edema improved compared with those before treatment, and the NYHA cardiac function classification improved by level 1. Ineffective: compared with the patients before treatment, the clinical symptoms and signs such as dyspnea, fatigue, and edema, and NYHA heart function classification did not improve or worsen compared with those before treatment.

(1) $$\begin{array}{c} \text{Total effective rate}=\frac{\left(\text{marked effect}+\text{effective}\right)}{\text{total number of cases}}\times 100\%\text{.} \end{array}$$

#### 2.3.2. Brachial Artery Endothelium-Dependent Vasodilation Function (EDD)

The baseline and follow-up examinations of all study subjects were performed by fixed ultrasound staff who had received uniform training. All patients were placed supine, had an empty stomach, rested for 30 minutes, and underwent color Doppler ultrasound examination. The upper arm was fully exposed, and the distance between the anterior and posterior intima of the brachial artery was recorded as the inner diameter (D0). Place a blood pressure cuff closer to the ultrasound probe and inflate it until the arterial systolic pressure is ≥ 30 mmHg. The arterial blood flow was blocked for about 5 minutes, then the cuff was quickly loosened to induce reactive hyperemia, and the inner diameter of the brachial artery (D1) was measured again after 1 minute of deflation.

(2) $$\begin{array}{c} \text{EDD}=\frac{\left(D1-D0\right)}{D0}\times 100\%. \end{array}$$

#### 2.3.3. Heart Function Test

All patients were tested by echocardiography (Shanghai Hanfei Medical Equipment Co., Ltd.). The changes of LVESD, LVEDD, CO, LVEF, and other indicators were observed before and after treatment in the two groups.

#### 2.3.4. NO and Endothelin (ET-1) Expression Level

In total, 4 mL of fasting venous blood was collected, and the levels of NO and ET-1 were measured by the nitrate reductase method and radioimmunoassay. The operation methods are strictly in accordance with the instructions. The above indicators were measured and recorded before and after treatment.

#### 2.3.5. Determination of Plasma NT-proBNP

An enzyme-linked immunosorbent assay (ELISA) method was used to collect 2 ml of fasting venous blood from the patient. The blood was placed in an anticoagulation test tube and a centrifuge with a rotation speed of 3000 r/min for 10 minutes of centrifugation was used. Plasma was separated and placed in a refrigerator at −20 °C overnight. The detection kit was provided by Wuhan Elabscience Biotechnology Co., Ltd. (E-EL-R3023). An automatic immunochemiluminescence instrument was used to detect plasma NT-proBNP levels. The correlation coefficient between NT-proBNP concentration and absorbance on the standard curve is > 0.995, indicating that the quality control parameters are within the standard error.

#### 2.3.6. Determination of APN and MMP-9 Levels

Serum adiponectin (APN) and matrix metalloproteinase-9 (MMP-9) levels were drawn on fasting before and after treatment. Enzyme-linked immunosorbent assay was used to detect the levels of APN and MMP-9 in the two groups before and after treatment.

### 2.4. Statistical Methods

The detection index data of the two groups of patients are expressed as mean ± standard deviation (SD). SPSS22.0 statistical analysis software was used for processing. Differences between different groups were compared by analysis of variance or chi-square test, and data between the same groups were tested by *t*-test. *P* < 0.05 indicates that the difference is statistically significant. Each experiment was repeated three times.

## 3. Results

### 3.1. Baseline Characteristics of Patients

This study selected 60 patients with hypertension and chronic heart failure. There were 30 cases in the research group, including 21 male patients and 9 female patients, with an average age of 74.37 ± 3.5 years. There were 30 cases in the control group, including 19 males and 11 females, with an average age of 75.97 ± 3.72 years. In general data comparison, the two groups of patients are comparable, and the difference is not statistically significant (*P* > 0.05) (Table 1).

### 3.2. Comparison of Clinical Effective Rate of Treatment between the Two Groups of Patients

In the research group, 2 cases were ineffective, 22 cases were effective, and 6 cases were markedly effective. The total effective rate was 93.3% (28/30). In the control group, 5 cases were ineffective, 15 cases were effective, and 10 cases were markedly effective. The effective rate was 83.3% (25/30).

### 3.3. Comparison of EDD Function between the Two Groups of Patients before and after Treatment

The difference in D0 between the two groups of patients after treatment was not statistically significant. Compared with the control group, the D1 (5.30 ± 1.85) mm in the research group after treatment was significantly higher than before (4.58 ± 1.31) (*P* < 0.05). EDD (11.83 ± 2.81) mm after treatment in the research group was significantly higher than before treatment (9.23 ± 2.17) (*P* < 0.05), as shown in Figure 1.

### 3.4. Heart Function Test

Before treatment, there was no significant difference in the levels of LVEDD, LVESD, and LVEF between the two groups of patients (*P* > 0.05) (Table 2). After treatment, the levels of heart function indexes LVEDD and LVESD of the two groups of patients were lower than before treatment (*P* < 0.05), LVEF levels were higher than before treatment, and the improvement of the research group was better than that of the control group, and the difference was statistically significant (*P* < 0.05) (Table 2).

### 3.5. Comparison of Plasma NO and ET-1 Levels before and after Treatment in the Two Groups

Compared with the control group, the NO (97.03 ± 7.53 *μ*moL/L) of the research group after treatment was significantly higher than that before treatment (83.04 ± 6.64 *μ*moL). Compared with the control group, the ET-1 (42.32 ± 4.82 ng/L) of the research group after treatment was significantly higher than that before treatment (49.97 ± 5.43 ng/L) (Figure 2).

### 3.6. Determination of NT-proBNP, APN, and MMP-9 Levels before and after Treatment

By comparison, we found that the NT-proBNP level in the research group before treatment was 4858.82 ± 512.34 pg/ml, the control group was 4835.43 ± 496.76 pg/ml, and there was no statistical difference between the two groups. After treatment, the NT-proBNP level in the research group was 985.35 ± 312.38 pg/ml, and the control group was 1203.19 ± 304.23 pg/ml. After treatment, the levels of NT-proBNP in the two groups were reduced compared with the same group before treatment, and there was a statistical difference. After treatment, the NT-proBNP level of the research group was significantly lower than that of the control group, and there were significant differences, indicating that the improvement of the research group was more obvious than that of the control group (Figure 3(a)). It can be seen from Figures 3(b) and 3(c) that there was no statistically significant difference in the levels of serum APN and MMP-9 between the two groups before treatment (*P* > 0.05). After treatment, the serum APN of the two groups was higher than that before treatment, and the level of MMP-9 was lower than that before treatment, and the improvement of the treatment group was better than that of the control group (*P* < 0.05).

### 3.7. Comparison of Carotid Artery Intima-Media Thickness, Glomerular Filtration Rate, and Left Ventricular Ejection Fraction before and after Treatment between the Two Groups

The difference in carotid artery intima-media thickness, glomerular filtration rate, and left ventricular ejection fraction before and after treatment in the two groups was not statistically significant (*P* > 0.05) (Table 3).

## 4. Discussion

Chronic heart failure (CHF) is a clinical syndrome characterized by excessive activation of neuroendocrine hormones and ventricular remodeling [19]. Chronic heart failure is the main clinical manifestation of various causes of heart disease in the terminal stage, with high morbidity and mortality. The main drugs currently used to treat chronic heart failure include the traditional golden triangle, including *β*-receptor blockers, aldosterone receptor antagonists, and angiotensin-converting enzyme inhibitors (ACEI)/angiotensin receptor antagonists (ARB). Among them, ACEI/ARB and *β*-blockers can effectively reduce the mortality of patients and improve the prognosis of patients [20]. ACEI/ARB and *β*-blockers play a key role in chronic heart failure and improve the clinical course of the disease [21]. The cornerstone of the treatment of chronic heart failure is to inhibit the renin-angiotensin-aldosterone system (RAAS). In addition, inhibiting enkephalinase and increasing the level of the natriuretic peptide can also effectively inhibit the activation of the neuroendocrine system, and the combination of the two can better play a synergistic effect [22]. The new type of chronic heart failure treatment drug sacubitril valsartan is the only angiotensin receptor-enkephalinase inhibitor (ARNI) used in clinical treatment. Sacubitril valsartan has a dual mechanism of action: not only can it inhibit enkephalinase, but also it antagonize angiotensin II receptors and have stronger antiproliferative and antifibrotic effects on cardiomyocytes [10].

Sacubitril valsartan is a new type of medicine for treating heart failure, mainly including sacubitril and valsartan. Sacubitril is an enkephalinase inhibitor, and enkephalinase is a multifunctional zinc-dependent metalloprotease. Enkephalinase can inactivate some peptide hormones, including brain natriuretic peptide and bradykinin, vasodilator peptides, glucagon, substance P, neurotensin, and oxytocin [23]. Valsartan is an angiotensin receptor antagonist. The main effect of valsartan is to inhibit the activation of the renin-angiotensin-aldosterone system and improve the long-term prognosis of patients with heart failure. As a compound preparation, sacubitril valsartan can be used in heart failure with reduced ejection fraction, which can effectively improve myocardial remodeling, thereby effectively reducing the risk of cardiovascular death in patients with heart failure, the risk of heart failure hospitalization, and the risk of all-cause death, and significantly improve and improve the symptoms and quality of life of patients. Studies have shown that sacubitril valsartan is an antihypertensive drug [24–26]. Sacubitril valsartan has a highly selective inhibition of enkephalinase, blocks angiotensin receptors, and plays an important role in improving heart failure, reducing ejection fraction, and controlling blood pressure [15, 27, 28]. In the occurrence and development of CHF, its vascular endothelial dysfunction and the disease itself are mutually causal. Brachial artery EDD is currently used clinically to evaluate the endothelial function of the body [29]. ET-1 is currently recognized as the strongest arteriovenous vasoconstrictor peptide, which is mainly secreted by endothelial cells. ET-1 can regulate vascular tone and stimulate the proliferation of vascular smooth muscle. The secretion of ET-1 *in vivo* increases when cardiomyocytes are damaged. Studies have shown that its expression is closely related to the severity of heart failure [30, 31]. Endogenous NO can expand the tube, lower blood pressure and protect cardiomyocytes [32]. BNP is a polypeptide hormone secreted and synthesized by cardiomyocytes, and its content is very small in normal humans. When the heart load increases or the heart function is impaired, its plasma concentration increases. Therefore, BNP is a specific indicator for diagnosing chronic heart failure, and it has important clinical value in evaluating therapeutic efficacy and predicting prognosis. APN is a protective plasma hormone protein secreted by adipocytes. APN participates in the occurrence, development, and prognosis of chronic heart failure of coronary heart disease through mechanisms such as inhibiting vascular inflammation, inhibiting monocyte adhesion, and the formation of fibrous tissue plaques. Pathological ventricular remodeling is an important pathological change in cardiovascular diseases, and MMP-9 is the main protease involved in ventricular remodeling. Studies have shown that MMP-9 activity is related to the severity of coronary heart disease and chronic heart failure. The higher the serum content of MMP-9, the more serious the deterioration of heart function.

The research group selected valsartan capsules and sacubitril and valsartan sodium tablets for comprehensive treatment and nursing of chronic heart failure and hypertension. The results of the study showed that compared with the control group, which was treated with valsartan capsules alone, after treatment, the serum APN, EDD function, and NO levels of the two groups of patients were significantly higher than before treatment, and the levels of MMP-9, BNP, and ET-1 were lower than before treatment. The improvement of the study group was better than that of the control group (*P* < 0.05). The results show that sacubitril valsartan and valsartan can improve the levels of heart failure markers in patients with chronic heart failure to the greatest extent, protect cardiomyocytes, and delay the development of ventricular remodeling [33]. However, due to the limited number of patients participating in the study, the data have limitations.

In summary, the treatment of valsartan capsules and sacubitril and valsartan sodium tablets in patients with hypertensive CHF can improve the patient's vascular endothelial function, increase serum APN levels, reduce MMP-9 and BNP levels, and improve the treatment efficacy of patients, which is worthy of clinical application.

## Figures and Tables

**Figure 1:** Comparison of EDD function between two groups of patients before and after treatment. *Note.* Compared with before treatment: ^*∗*^*P* < 0.05; compared with the control group:  ^#^*P* < 0.05; (a) D0, (b) D1, and (c) EDD.

**Figure 2:** Comparison of plasma NO and ET-1 levels before and after treatment in the two groups. (a) NO level and (b) ET-1 level.

**Figure 3:** Comparison of NT-pro BNPAPN and MMP-9 levels before and after treatment in the two groups. *Note.* (a) Level of NT-pro BNP, (b) level of APN, and (c) level of MMP-9.

**Table 1:** Comparison of general information.

Project	Research group	Control group	*t*/*x*^2^	*P*
Gender (male/female)	21/9	19/11	0.3	0.58
Age (year)	74.37 ± 3.5	75.97 ± 3.72	1.71	0.09
Mean arterial pressure (mmHg)	130.21 ± 10.98	128.45 ± 11.15	0.62	0.54
BMI (kg/m^2^)	31.23 ± 4.01	30.11 ± 4.25	1.06	0.29

**Table 2:** Comparison of echocardiographic indicators before and after treatment between the two groups.

Time	Index	Control group	Research group	t value	*P* value
Before treatment	LVEDD (mm)	61.21 ± 9.14	62.76 ± 9.32	0.65	0.52
	LVESD (mm)	41.89 ± 7.14	42.31 ± 7.99	0.21	0.83
	LVEF (%)	31.32 ± 4.96	30.04 ± 5.03	0.99	0.32
After treatment	LVEDD (mm)	57.79 ± 6.87	54.87 ± 6.45	1.70	0.09
	LVESD (mm)	37.85 ± 5.42	34.36 ± 5.04	2.58	0.01
	LVEF (%)	34.48 ± 4.52	36.88 ± 5.02	0.99	0.32

**Table 3:** Comparison of carotid artery intima-media thickness before and after treatment between the two groups of patients, glomerular filtration rate, and left ventricular ejection fraction.

Group	Carotid artery intima-media thickness (mm)			Glomerular filtration rate (ml/min)			Left ventricular ejection fraction (%)		
	Before treatment	After treatment	Difference	Before treatment	After treatment	Difference	Before treatment	After treatment	Difference
Control group	1.23 ± 0.22	1.28 ± 0.24	0.05 ± 0.07	123.45 ± 19.35	118.75 ± 16.36	−3.11 ± 7.35	39.39 ± 1.81	41.22 ± 2.08	1.83 ± 0.66
Research group	1.24 ± 0.21	1.30 ± 0.26	0.05 ± 0.09	122.33 ± 19.14	121.86 ± 17.83	−0.47 ± 5.15	39.02 ± 1.73	41.44 ± 2.11	2.42 ± 0.73

## Data Availability

The data to used support the findings of this study are available on reasonable request from the corresponding author.
